This article has been retracted.

# A Multicenter Cohort Study on Children Suffering from Acute Lymphoblastic Leukemia: Effects of Obesity on Mortality

**DOI:** 10.1155/2022/4880151

**Published:** 2022-07-05

**Authors:** Xiangwen Wang, Dan Mu, Anyang Geng, Anqi Zhao, Yiyuan Song

**Affiliations:** ^1^Inner Mongolia International Mongolian Hospital, Hohhot, China; ^2^Inner Mongolia People's Hospital Pediatric Hematology, China

## Abstract

**Background:**

Overweight and obesity have been reported in specific patients and disease survivors compared to other types of childhood cancer. This study is aimed at determining the effect of children's obesity on the mortality of acute lymphoblastic leukemia.

**Method:**

Children admitted to Inner Mongolia International Mongolian Hospital from 1 January 2017 to 31 December 2020 participated in this study. 1070 children were analyzed. A multi-middle-class poll was conducted. All children under the age of 15 were followed up within 24 months of diagnosis. Overweight and obesity are identified according to the World Health Organization and the Centers for Disease Control and Prevention. Premature death and reoccurrence of emergencies are the main consequences.

**Results:**

The initial ethical rate for the first 24 months of testing was 19.9% (NS 213). The lowest cancer survival rate (DFS) was childhood obesity (73%) (24 months), compared with average weight (81%). Diagnosis of overweight/obesity is a predictor of early death (WHO: HR = 1.4, 95% CI: 1.0-2.0; CDC: HR = 1.6, 95% CI: 1.1-2.3). However, there was no association between overweight and obesity (WHO: HR = 1.5, 95% effective interval: 0.9-2.5; CDC: human resources = 1.0, 95% effective interval: 0.6-1.6) and obesity (WHO: HR = 1.5, 95% effective interval: 0.7-3.2; CDC: HR = 1.4, 95% effective interval: 0.9-2.3). Early recurrence was observed.

**Conclusion:**

Overweight and obese people belong to the subclass with a high risk of death in the treatment of leukemia.

## 1. Introduction

China has one of the highest child leukemia mortality rates in the world. Despite reluctance to undergo chemotherapy in similar countries, mortality rates have increased in recent years through early treatment [1].

In some countries, the rate excluding morgues is about 1-2 percent. However, Honduras (20.8 percent), Brazil (14.9 percent), and India (1.7 percent) reported very high mortality rates in developing countries during this healing process. In China, Luna et al. also reported mortality at the time of introduction (15%), and early decline has been found to be a major obstacle to improving survival rates among Chinese children. This is a higher incidence in countries (3-4.5 percent) (17-22.1 percent). Importantly, it has been shown that both overweight and obesity are associated with a high risk of child recovery and death [2, 3].

There are many hypotheses that explain the sensitivity of overweight and obese patients to rest and the inability to receive chemotherapy. As a result, high cholesterol levels have been shown to contain leukemia cells rather than being protected by chemotherapy nearby [4].

To date, a number of international studies have been carried out to examine the social weight and obesity rates, as well as the rates of decline and survival, in all children. Based on the body mass index (BMI) and age and gender nutrition data from the CDC and WHO, the evidence sheet has been widely used to assess these nutritional changes [5]. The authors have yet to agree on the effects of BMI drugs, toxic chemotherapy, and chemotherapy effects.

Considering that overweight and obesity in China, as well as mortality from prostate cancer in children, have been increasing for many years and considering that nutrition may be a factor, the purpose of this study is to study whether weight and obesity can lead to premature falls and deaths in our people [6].

## 2. Methods

The institute (MIGICCL) conducted a series of tests at hospitals to determine the cause of leukemia in China. Between 1 January 2017 and 31 December 2020, any participants in the hospital were children. Children downtown and nonresidents of Beijing are discriminated against. Each child is 24 months after diagnosis [7].

Participating institutions include the China Social Security Association, the Director General of the Social Security Bureau, and the China Institute of Indigenous Security Department of Social Security and Social Services (ISSSTE). All customers are treated in their healthcare system according to their chemotherapy diet [8]. Our study was approved by the institutional review board of the hospital and was conducted in accordance with the ethical principles originating from the Declaration of Helsinki.

During the study period, a total of 1254 children were diagnosed with short-term leukemia in participating hospitals. Of these, 26 (2.1%) Inuit declined and 113 (9%) were unable to follow up because they did not live in Beijing, and the weight and level of 45 children were not found in their health records. The inclusion criterion was patients diagnosed with leukemia. The exclusion criterion was that patients received the chemical and radioactive treatment.

### 2.1. Data Purchases

Information on age, gender, habitat, list of white blood cells, immune system type (B or T), weight and height (appropriate), and chemotherapy diet were recently compiled by the patient's medical records for staff standards—Bronfman standards (high SES, up to 1.5 people per bedroom; low SES and medium SES, each with more than 1.6 people per bedroom), and coastal areas are used as advocates for socioeconomic conditions (SES). The risk rating is based on the National Cancer Institute (NCI) standard: common hazards (age 9.99; white blood cell count < 50 × 10^9^/L) or high risk (age < 1and >10 years old or WBC > 50 × 10^9^/L). In this study, the first death was confirmed as the patient at any time within 24 months of diagnosis. The first reemergence of bone markers has been confirmed, as patients rapidly had >25% from the bone marrow for the first time since the bone marrow exploded. The general anxiety system (CNS) is designed to be present in body fluids with a short color (CSF) in cells that use the first CR, and a count is 5/mL or uncolored [9].

### 2.2. Nutritional Status Analysis When Complex Leukemia Is Found

Use BMI to evaluate. Using PC software ThroPlus (Table 3.2.2, WHO, Geneva), calculate the number of infants per patient. According to the people they identified, patients were classified as regularly used (-1.9999-0.9999), waste (-2-2.9999), waste (>-3), weight (1-1.9999), overweight (2-2.9999), and obesity (>3). In addition, CDC gives BMI% reduction: general (p5-84.9999), weight (<p5), weight (p85-94.9999), and obesity (>p95). For nutritional characteristics and measurements, as described in this survey, weight and grade data from clinical data are used to determine the nutritional status of patients.

### 2.3. Statistical Analysis

For data analysis, see SPSS Section 21 (IBM). Calculate the 95% confidence interval (CI) for detailed data and vulnerabilities (RRs). Family planning survival tests were conducted in the early stages of crashes and early deaths. The incoming inspection is counted. The studies were conducted independently in the early fall or early death, adjusting previous records of the various information (age, gender, HIV, NCI risk identification, and chemotherapy) that influenced the results [10].

Using the results of the relevant studies, they were found to be significantly associated with (0.74) age and NCI risk. Therefore, the decision to delete different age groups in the system is not discussed. Therefore, the shortest examples include gender, SES, vaccine, NCI risk levels, chemotherapy, and nutritional status. The Cox thrusters are dangerous substances. Risk (HR) is 95% CI forecast. In addition, the Cox isolation assessment, by the age group and NCI risk level, has been adjusted to accommodate differences within the system [11].

## 3. Results

### 3.1. General Information

According to the World Health Organization, 61.5 percent (NS 658) weighs 18.4 percent of tons (NS 197), 8.9 percent (NS 95) is determined to be weighted, and 4.2 percent (NS 45) is classified as obese. According to the code, 13% (NS 129) is diabetes and 14.1% (NS 140) is diabetes. The majority of patients identified as weighted by the World Health Organization (92%) also met CDC obesity guidelines (Table 2). Between 18 and 24 months, a total of 160 cases (15 percent) were initially raised between 6 [6] and 20 (12.5 percent), including bones (66.9%; *n* = 107) and beyond [12].

### 3.2. Individual Anxiety System Recovery (NS 32; 20%)

The initial ethical rate for the first 24 months of testing was 19.9% (NS 213). Of these, 148 (69.5 percent) were initially processed. The main causes of death are as follows: risk (NS 141; 66.4%), risk (NS 30; 13.9%), and leukemia activity (NS 24; 11.3%). The risk of repetition and death in childhood of <1 year and >10 years is shown in Table 2.

The lowest cancer survival rate (DFS) was childhood obesity (73%) (24 months), compared with average weight (81%) (Figure 1). Although average weight/excessive weight is used to determine the nature of the condition, the Department of Family Services has a lower level of knowledge of the obesity group, which was less accurate (form) (*P* = 0.07) (Figure 1).

### 3.3. Obesity Was Associated with Lower Child Survival Rates

Obesity (68%) was shown to have lower child survival rates, with OS (75%) slightly higher than the patient's weight. There are differences between Somali patients and overweight patients when diagnosed at the same time (Expert Group), compared to childhood obesity (Figure 2). By reference to differences and RR-related risks, the 95% confidence gap is more pronounced (digital level; *P* = 0.003) (Figure 3).

For children and children who may be overweight, the number of social service workers is 80 percent and 81 percent, respectively. In contrast, children with lower levels of weight (71 percent) and obesity (73 percent) have lower rates of social services. The Department of Family Services is lower than the weight/obesity group (72 percent) (81 percent) but less accurate (Clinton; *P* = 0.06) (Figure 4).

In the Cox model, the results showed that overweight and obesity were associated with an increased risk at the beginning of the new period, but the confidence gap was wrong (HR: 1.5, 95% CI: 0.9-2.5 and HR: 1.5, 95% CI: 0.7-3.2; various). Subsequently, on a case-by-case basis, secondary weight loss and obesity in children were associated with short periods of time, taking into account the average weight and weight status of the patients. However, the confidence gap is accurate (HR: 1.4, 95% CI: 0.9-2.2).

### 3.4. Weight Is Associated with an Increased Risk of Premature Death

It should be noted that overweight and obese patients are underweight (68% and 70%) (OS: 80%). OS is 75%, slightly higher than for people who are overweight or obese (upcoming *P* = 0.04) [13]. In determining average weight and weight loss risk, the gap in OS was higher than that in patient contacts over 24 months, as well as in patients who were overweight and obese as partners (document; *P* = 0.01) (Figure 5).

Weight is associated with an increased risk of premature death (HR: 1.5, 95% CI: 1.0-2.3), but obesity is as determined (HR: 1.5, 95% confidence gap: 0.8-2.7). Therefore, reconsider the differences in exposure (overweight/obesity group, high risk of early death) (HR: 1.4, 95% CI: 1.0-2.0) [14].

### 3.5. Weight Is Associated with Early Death

Associated weight/obesity and early death were assessed as high as NCI risk. Similar findings have been observed in other room risks (HR: 1.5, 95% CI: 0.7-2.9) and high risk (HR: 1.5, 95% CI: 0.9-2.3).

In addition, by age, the risk of early death due to obesity is higher than >10 (HR: 2.0, 95% CI: 1.2-3.3) and 1-9.9 years (HR: 1.2, 95% CI: 0.7-2.2). Importantly, if all infants (<1 year old) are excluded from the assessment, the risk will not change [15].

## 4. Discussion

China has one of the highest rates of leukemia in the world, but child mortality has not decreased in recent years. In addition, Latin America is the country that has survived the most since Ecuador. In previous studies, it was reported that there were differences in clinical conditions in all patients in China compared to children in other survival groups. For example, according to NCI standards, about 50 percent of Chinese children are classified as high-risk recaptures, and ETV6-RUNX1 (7 percent) can be found in children with fewer parents whose genetic code is associated with the original disease. Alternatively, one-third of patients in these countries are diagnosed with a high risk of recurrence, and 22% of ETV6-RUNX1 has been diagnosed [14].

As far as we know, this study is the first to explore the relationship between overweight, obesity, and child mortality, as well as all the risks of reemergence in China. In the first 24 months of diagnosis, the average fatal disease was 19.9%. In particular, the mortality rate is considered to be very high in the first two months of the study, and keep in mind that the follow-up of all children in the country (approximately 6.8%) is developing [16].

In fact, overweight and obesity have been reported in specific patients and disease survivors compared to other types of childhood cancer. Specifically, all child archeologists showed the highest levels of weight and obesity in care. In other populations, with similar results to this study, the presence of overweight and obesity is associated with symptom elimination and survival. In another Cox study, the organization was observed to be overweight and at risk of premature death. Nevertheless, confidence in the weight and premature death gap is accurate. In another study, the link between obesity and early death was assessed at higher levels of NCI by showing that children's weight could be exposed. Similar findings have been observed in other room risks (HR: 1.6, 95% CI: 0.8-3.1) and high risk (HR: 1.7, 95% CI: 1.1-2.7). Another age study showed that obese patients had a higher risk of obese children at age 10 (HR: 2.1, 95% CI: 1.3-3.5) and 1-9.9 years (HR: 1.2, 95% CI: 0.6-2.2).

Orgel et al.'s meta-analysis study showed that children had the highest risk of weight loss/obesity death in 11 tests (HR: 1.3, 95% CI: 1.1-1.6). In another study by Amono et al., a link was also shown between obesity and overweight and obesity over the next five years (HR: 1.3, 95% CI: 1.2-1.5). The findings are similar to those discussed by other researchers. In contrast, this error is associated with obesity and low survival rates (HR: 1.4, 95% CI: 0.69-2.87), which are listed in the patient's combination of archeologically specific mumps [17].

In the current study, both CDC 2000 and economic data were used to determine the nutritional status of the introduction of BMI. BMI is reported to be directly related to body fat measurements (skin thickness, natural ultrasound, two-sided energy radiation, and other methods of richness). Thus, these two specific indicators indicate the results obtained from the current survey and may be higher [18].

The average weight of the Centers for Disease Control and Prevention (27.1 percent) and WHO (13 percent) has been lower than that of all children in other populations using various nutritional levels, such as the United Kingdom (35 percent, IOTF), Brazil (35.9 percent, WHO), and Canada (33.2 percent, CDC). However, the CDC outbreak is the same as the outbreak in all children in Malaysia, China, and India (24.5%, WHO).

On the other hand, the average initial reemergence rate in this survey was 14.9 percent, lower than the three previously reported by Zimmerman-Hernandez et al. in three public hospitals in China (22.1 percent) and Ontario to Guatemala (14.9 percent) but similar in most countries (<5 percent). The results of the study revealed collaborations on obesity or obesity risk to ensure the accuracy of statistics. Previous studies have reevaluated the relationship between weight and obesity and overweight and obesity and risk over the past five years, with different results. For example, from studies conducted by Ankara et al., studies showed childhood obesity (HR: 0.73, 95% CI: 0.59-0.91), and another study showed a higher risk (HR: 1.29, 95% CI: 1.02-1.56). In a study conducted by Gelete et al., they reported a high risk of recurrence of various aspects of childhood obesity during the five-year follow-up period (HR: 1.3, 95% CI: 1.0-1.6). Alternatively, Apple and others surveyed 768 children and found that they had a lower risk of obesity than children who lost an average weight (HR: 0.7, 95% CI: 0.6-0.9) [19].

One possible reason for the error estimate is that the potential additional risk in this study is the low abundance generated during the study period. It is therefore important to maintain this record over the next three years to assess the relationship between the nutritional changes and the average number of all children in China [20].

Currently, chemotherapy drugs are at the top of the child's weight and/or the patient's body. So far, there is no evidence that the most suitable patients to adjust for medication and stress require chemotherapy for weight and obesity. This may cause the patient to receive oxygen pills, which increases the risk of toxins or reemergence [21].

Given the results of this exercise and recently reported social overweight and obesity, as well as being potentially fatal, additional treatment should be considered for overweight/obese children [22], so the risk of serious problems associated with obesity, chemotherapy, and increased support requires tissue therapy programs, such as those that survive the most [23, 24].

## 5. Conclusion

In China, overweight and obesity are separate from predicted mumps deaths in children [25]. Monitoring these children will improve their survival rate. Importantly, more research is needed to better understand biological movements associated with overweight and obesity in response to drug abuse and toxins [26].

## Figures and Tables

**Figure 1:** Disease-free survival (early relapses) according to CDC 2000 nutritional classification (three categories).

**Figure 2:** Disease-free survival (early relapses) according to CDC 2000 (two categories).

**Figure 3:** Overall survival up to 24 months according to CDC nutritional status.

**Figure 4:** Disease-free survival (early relapses) according to WHO nutritional classification.

**Figure 5:** Overall survival up to 24 months after diagnosis according to WHO nutritional classification.

**Table 1:** Clinical status of patients diagnosed in health centers between 2017 and 2020.

Transition	Predator *n* (%) 1254 (100)	Examine		Handkerchief
		He is right *n* (%) 1070 (85.3)	No, sir *n* (%) 184 (14.7)	
Male-female body movements				
	684 (54.5)	595 (55.6)	89 (48.4)	0.07
Female	570 (45.5)	475 (44.4)	95 (51.6)	
Fiscal year (year)				
<1	34 (2.7)	28 (2.6)	6 (3.3)	0.29
1-9.9	840 (67.0)	726 (67.9)	114 (62.0)	
>10	380 (30.3)	316 (29.5)	64 (38.8)	
Socioeconomic status				
Medium to low	1043 (85.2)	902 (85.7)	141 (82.0)	0.20
Quttiktuq	181 (14.8)	150 (14.3)	31 (18.0)	
Introduction of the white blood cell count (×10^9^/L)				
<10	605 (48.2)	526 (49.2)	79 (42.9)	0.18
10-49.99	373 (29.7)	306 (28.6)	67 (36.4)	
50~99.99	107 (8.5)	91 (8.5)	16 (8.7)	
>100	169 (13.5)	147 (13.7)	22 (12.0)	
NCI risk level				
Standard 2	691 (55.1)	597 (55.8)	94 (51.1)	0.24
Quttiktuq	563 (44.9)	473 (44.2)	90 (48.9)	
Immune system				
Introduction to the B-level course	1077 (85.9)	915 (85.5)	162 (88.0)	0.60
Aging	20 (1.6)	16 (1.5)	4 (2.2)	
Dual phenoform	42 (3.3)	37 (3.5)	5 (2.7)	
T cells	115 (9.2)	102 (9.5)	13 (7.1)	

Captain Pearson.

**Table 2:** Two factors that first relapse and die early in the first 24 months of diagnosis.

Transition	Quick fall			Untimely death		
	Activity	Moratorium	Increase muscle by 95%	Activity	Moratorium	Increase muscle by 95%
Male and female body movements						
Female (code)	54	1	—	103	1	—
Man	106	1.7	1.2-2.4	110	0.8	0.6-1.1
Age						
1-9.9 years (contact)	92	1	—	111	1	—
<1 year	8	2.7	1.2-6.4	15	6.4	2.9-13.8
>10 years	60	1.6	1.1-2.3	87	2.1	1.5-2.9
NCI risk level						
Standard (contact information)	66	1	—	81	1	—
Quttiktuq	94	1.9	1.4-2.8	132	2.5	1.8-3.3
Immune system						
Employment front (contact information)	138	1	—	173	1	—
Aging	4	1.8	0.6-5.9	3	0.9	0.3-3.5
Dual phenoform	5	0.8	0.3-2.3	7	1.0	0.4-2.3
T cells	13	0.8	0.4-1.5	30	1.8	1.1-2.8
Socioeconomic status						
High (contact information)	32	1	—	32	1	—
Mild nutritional status	127	0.6	0.4-0.9	173	0.9	0.6-1.3
Centralized health and intervention programs (%)						
General (p5-84.9) (contact information)	79	1	—	95	1	—
Weight (p85-94.9)	19	1.1	0.6-1.9	29	1.5	0.9-2.4
Obesity (>p95)	25	1.4	0.8-2.2	39	1.9	1.3-3.0
World Health Organization (Z-class)						
General (-1.9-0.9) (contact information)	96	1	—	118	1	—
Overweight (1-1.9)	28	0.9	0.6-1.5	45	1.4	0.9-2.0
Weight (2-2.9)	18	1.4	0.8-2.4	25	1.6	1.0-2.7
Obesity (>3)	8	1.3	0.6-2.8	12	1.7	0.8-3.3

## Data Availability

The data used to support this study is available from the corresponding author upon request.
